The article "Ailanthone Induces Cell Cycle Arrest and Apoptosis in Melanoma B16 and A375 Cells" was retracted in 2020. Reason: duplicated images.

# Ailanthone Induces Cell Cycle Arrest and Apoptosis in Melanoma B16 and A375 Cells

**DOI:** 10.3390/biom9070275

**Published:** 2019-07-11

**Authors:** Wenjing Liu, Xiaona Liu, Zhaohai Pan, Dan Wang, Minjing Li, Xiaoyu Chen, Ling Zhou, Maolei Xu, Defang Li, Qiusheng Zheng

**Affiliations:** 1 Yantai Key Laboratory of Pharmacology of Traditional Chinese Medicine in Tumor Metabolism, School of Integrated Traditional Chinese and Western Medicine, Binzhou Medical University, Yantai 264003, Shandong, China; 2 School of Pharmacy, Binzhou Medical University, Yantai 264003, Shandong, China

**Keywords:** ailanthone, cell cycle arrest, cell apoptosis, B16 cells, A375 cells mitochondria

## Abstract

Malignant melanoma is the most lethal type of skin cancer. Previous studies have shown that ailanthone has potent antitumor activity in a variety of cell lines. However, the anti-tumor effect of ailanthone on malignant melanoma remains unclear. To investigate the anti-tumor mechanisms of ailanthone in human melanoma B16 and mouse melanoma A375 cells, the cell counting kit-8 assay, colony formation assay, DNA content analysis, Hoechst 33258, and Annexin V-FITC/PI staining were used to assess cell proliferation, cell cycle distribution, and cell apoptosis, respectively. Western blotting was performed to evaluate the expression of cell cycle- and apoptosis-related proteins and regulatory molecules. The results showed that ailanthone significantly inhibited melanoma B16 and A375 cell proliferation as well as remarkably induced cell cycle arrest at the G0–G1 phase in B16 cells and the G2–M phase in A375 cells in a dose-dependent manner. Further investigation revealed that ailanthone promoted the expression of p21 and suppressed the expression of cyclin E in B16 cells or cyclin B in A375 cells through the PI3K-Akt signaling pathway. In addition, ailanthone induced B16 and A375 cell apoptosis via a caspase-dependent mechanism. Further studies showed that ailanthone remarkably downregulated Bcl-2 and upregulated Apaf-1 and Bax, and subsequently increased mitochondrial membrane permeabilization and released cytochrome c from the mitochondria in B16 cells and A375 cells. Taken together, ailanthone induces cell cycle arrest via the PI3K-Akt signaling pathway as well as cell apoptosis via the mitochondria-mediated apoptotic signaling pathway. Ailanthone may be potentially utilized as an anti-tumor agent in the management of malignant melanoma.

## 1. Introduction

Malignant melanoma is the most lethal type of skin cancer. Its five-year survival rate is less than 10%, prognosis is often extremely poor, and its incidence and mortality are higher than any other tumor type [1]. It is highly invasive, blood and lymphatic vessel metastasis can occur during the early stage of tumor formation, and is thus one of the most malignant tumors that seriously threaten human health [2]. In recent years, in addition to traditional surgical treatment, anticancer therapy has improved, which includes the use of targeted therapy and immunotherapy [3]. However, despite higher patient response rates using targeted therapy and immunotherapy, the long-term survival rate of malignant melanoma remains very low [4] and is also prone to drug resistance in the later stage of treatment. A few effective low-toxicity drugs have been used in the treatment of cancer [5]. Therefore, the development of more effective treatment schemes for melanoma is essential [6].

Medicinal plants have historically been used in the treatment of various cancers [7]. Many Asian countries including China, Japan, and Thailand have used traditional medical phytotherapy for cancer treatment for thousands of years [8]. Several current clinical anticancer drugs such as paclitaxel and vinblastine are also derived from plant extracts. Plants are thus major resources for new anticancer drugs [9]. In addition, plant-derived drugs exhibit fewer side effects than chemical drugs [10]. Therefore, there is increasing interest in identifying and isolating natural compounds from medicinal plants in order to develop new anticancer drugs and improve the reactivity and long-term survival of cancer patients.

Ailanthone (as shown in Figure 1), extracted from the traditional Chinese plant *Ailanthus altissima* [11], has been reported to have anti-tuberculosis, anti-viral, and anti-tumor activities [12]. A study reported that ailanthone could be used as a novel drug for the treatment of prostate cancer [13]. Ailanthone can also significantly inhibit non-small cell lung cancer migration, invasion, and metastasis, indicating its potential as a novel treatment regimen [14]. Moreover, ailanthone inhibits the proliferation of gastric cancer SGC7901 cells and induces cell cycle arrest at the G2/M phase [15,16]. In addition, ailanthone can also cause autophagy, apoptosis, and cell cycle arrest at the G0/G1 phase in human promyelocytic leukemia HL-60 cells [17]. These findings confirm that ailanthone has anti-tumor properties, although its effect on malignant melanoma and its mechanism of action remain unclear. Therefore, this study used melanoma B16 and A375 cells to evaluate the anti-tumor effect of ailanthone.

## 2. Materials and Methods

### 2.1. Cell Lines and Culture Conditions

Human melanoma A375 cells (Cat no. SCSP-533) and mouse melanoma B16 cells (Cat no. TCM 2) were obtained from the Cell Bank of Type Culture Collection of Chinese Academy of Sciences China (Shanghai, China). The cells were cultured in a sterile cell culture chamber (HF240, HEALFORCE, Shanghai Lishen Scientific Equipment Co. Ltd.) with 95% air and 5% CO_2_ saturated humidity at a temperature of 37 °C. Human melanoma A375 cells were subsequently cultured and tested using DMEM high glucose medium (Cat no. SH30022.01, Hyclone) supplemented with 10% FBS (Cat no. 10091-148, Gibco), 1% streptomycin mixture (Cat no. P1400, Solarbio), and 1% sodium pyruvate (Cat no. SP0100, Solarbio). Mouse B16 cells were cultured in 1640 medium (Cat no. SH30809.01, Hyclone) supplemented with 10% FBS and 1% streptomycin mixture.

### 2.2. Cell Proliferation Assay

The cultured B16 and A375 cells were trypsinized and collected by centrifugation at 800× *g* for 3 min and seeded into 96-well plates at a density of 8 × 10^3^/well and cultured overnight. Ailanthone (Cat no. SA9130, purity: ≥98%) was purchased from Solarbio Life Sciences (Beijing, China). Different concentrations of ailanthone (0.25, 0.5, 1, 2, 4, 8, and 16 μM) in DMSO were added to each well (*n* = 3 for each concentration) and a solvent control group was set up. The 96-well plate was then placed in a cell culture incubator for 24 h. Then, 100 μL of a CCK-8 solution (Cat no. CK04, Dojindo) were added to each well and further cultured for 2 h in an incubator. Then, the absorbance of each well was measured at a wavelength of 450 nm using a multi-plate reader (Infinite 200 PRO, Tecan, Tecan Austria GmbH, Untersbergstrasse 1a, A-5082 Grödlg, Austria), and the proliferation inhibition rate of the B16 and A375 cells in the presence of different concentrations of ailanthone was calculated [18].

### 2.3. Colony Formation Assay

Cells (density: 1.5 × 10^2^ cells/well) were seeded into six-well plates and incubated overnight. Then, different concentrations of ailanthone were added to each well and the cells were cultured for another 24 h. The cells were then maintained in fresh medium for 14 days. The obtained colonies were fixed with a 4% tissue fixing solution (Cat no. P1110, Solarbio) for 20 min and then stained with 1% crystal violet (Cat no. G1062, Solarbio) for 15 min. The number of colonies with a diameter >0.5 mm was counted under an inverted microscope (Leica DMI3000B, Leica Microsystems CMS GmbH, Wetzlar, Germany).

### 2.4. Hoechst 33258 Staining

Cells at the logarithmic growth phase were harvested using 0.25% trypsin and centrifuging at 800× *g* for 3 min to collect the cells. The cells were seeded into a six-well plate at a density of 2 × 10^5^ cells/well. After incubating for 24 h at 37 °C and 5% CO_2_ incubator, different concentrations of ailanthone were added, and the cells were further cultured for another 24 h in the incubator. After incubation, the cells were stained, and cell morphology was assessed under a fluorescence microscope (DMI3000B, Leica, Leica Microsystems CMS GmbH) [19].

### 2.5. Apoptosis Detection by Annexin V-FITC/PI Staining

Cells (2 × 10^5^/well) were seeded into six-well plates and grown overnight, then exposed to different concentrations of ailanthone for 24 h. Cells were then carefully collected and analyzed for reaction with annexin V-FITC/PI (Cat no. CA1020, Solarbio) according to the kit instructions (Beijing Solarbio Science & Technology Co., Ltd., Beijing, China), and the green fluorescence from annexin V-FITC and red fluorescence from PI were analyzed using flow cytometry (FACSCanto II, Becton, Dickinson and Company, New Jersey, USA) [19].

### 2.6. DNA Content Analysis

The cells (2 × 10^5^/well) were seeded into six-well plates and incubated overnight at 37 °C in a 5% CO_2_ incubator before treatment with different concentrations of ailanthone for 24 h. The cells were then collected and fixed in 75% ethanol at −4 °C overnight, incubated with 50 ng/mL PI staining solution and 0.1 mg/mL RNase A (Cat no. CA1510, Solarbio) for 30 min in the dark at 37 °C, and finally analyzed for DNA content by flow cytometry [20].

### 2.7. Mitochondrial Membrane Potential Measurement

Cells (2 × 10^5^/well) were seeded into six-well plates and grown overnight, after ailanthone treatment for 24 h. JC-1, at a concentration of 10 μg/mL, was added to the medium for 20 min. The cells were then washed twice in JC-1 staining buffer (Cat no. M8650, Solarbio). Fluorescence emission was detected at wavelengths of 529 and 590 nm. The change of mitochondrial membrane potential in ailanthone-treated cells was observed under a fluorescence microscope [21].

### 2.8. Western Blot Analysis

Cells (2 × 10^6^/Petri dish) were inoculated into 100 mm culture dishes and grown overnight, and then incubated with different concentrations of ailanthone for 24 h. After treatment, the cells were harvested and lysed on ice for 30 min in RIPA buffer (Cat no. R0010, Solarbio) containing 0.1 M PMSF and a mixture of the protease and phosphatase inhibitor. The lysate was centrifuged at 12,000× *g* for 15 min at 4 °C, and the supernatant was collected and stored at −80 °C. Cell lysates (80 μg) were separated by SDS-PAGE, transferred to PVDF membranes (Cat no. ISEQ00010, Millipore, Burlington, USA), blocked with 5% milk, and probed with primary antibodies (β-actin, Cat no. TA-09, 1:2000, ZSGB-Bio; PI3K, Cat no. ab19606, 1:1000, Abcam; p-PI3K, Cat no. ab182651, 1:1000, Abcam; Akt, Cat no. ab8805, 1:500, Abcam; p-AKT, Cat no. ab38449, 1:1000, Abcam; p21, Cat no. ab109199, 1:1000, Abcam; Cyclin B, Cat no. ab32053, 1:1000, Abcam; Cyclin E, Cat no. ab194070, 1:5000, Abcam; Caspase-3, Cat no. ab13847, 1:1000, Abcam; Cleaved Caspase-3, Cat no. ab49822, 1:500, Abcam; Caspase-9, Cat no. 9508S, 1:1000, Cell Signaling Technology; Cleaved Caspase-9, Cat no. E5Z7N, 1:1000, Cell Signaling Technology; Apaf-1, Cat no. R205, 1:1000, Cell Signaling Technology; Cyt C, Cat no. 136F3, 1:1000, Cell Signaling Technology; Bcl-2, Cat no. ab196495, 1:1000, Abcam; or Bax, Cat no. ab182734, 1:1000, Abcam) and appropriate secondary antibodies (peroxidase-conjugated goat anti-mouse IgG (H + L), Cat no. ZB-2305, 1:50,000, ZSGB-Bio; or goat anti-rabbit IgG H&L, Cat. no. ab6721, 1:20,000; Abcam). The immunoreactive bands were visualized with a developer using a gel imaging analysis system (BioSpectrum 510 Imaging System Motorized Platform, UVP, UVP/Analytik Jena, Jena, Germany) [22].

### 2.9. Statistical Analysis

The results were expressed as means ± standard deviation (SD). The difference between groups was analyzed by GraphPad Prism 6.0 software. The student’s *t* test or one-way ANOVA were used to calculate the statistical difference, and *p* < 0.05 was considered statistically significant.

## 3. Results

### 3.1. Ailanthone Inhibits Cell Proliferation and Colony Formation in Melanoma B16 and A375 cells

We first evaluated the anti-tumor effects of ailanthone on melanoma cells using a cell counting kit-8 assay in both mouse B16 and human A375 melanoma cells. Cells were treated with different concentrations of ailanthone (0.25, 0.5, 1, 2, 4, 8, and 16 μM) for 24 h. The results indicated that ailanthone significantly decreased the cell viability of both B16 and A375 cells in a concentration-dependent manner, with the IC_50_ values of 1.83 and 5.77 μM, respectively (Figure 2a). Moreover, we assessed the effect of ailanthone on the cell colony formation of melanoma cells. Depending on the results of the assay, treatment with different concentrations of ailanthone induced a dose-dependent decrease in the number of B16 and A375 cell colonies (Figure 2b,c).

### 3.2. Ailanthone Induces Melanoma Cell Cycle Arrest and Regulates the Levels of Cell Cycle-Related Proteins in Melanoma B16 and A375 Cells

To determine the possible intrinsic mechanism of ailanthone-induced melanoma cell proliferation inhibition, we measured the cell cycle phase distribution of ailanthone-treated cells by flow cytometry with propidium iodide (PI) staining. We found that ailanthone treatment induced G0/G1 phase accumulation in B16 cells when compared to the control group (Figure 3a,b). To investigate the mechanism of ailanthone on cell cycle arrest in B16 cells, the expression levels of cell cycle-related proteins (e.g., p21, cyclin B, and cyclin E) were examined by Western blotting. The results showed that ailanthone treatment caused an increase in the expression level of p21 and a decrease in cyclin E expression in B16 cells (Figure 3c,d). Similarly, we found that ailanthone induced significant G2/M phase arrest in A375 cells when compared to the control group (Figure 3e,f). Ailanthone treatment also induced an increase in the expression level of p21 and a decrease in cyclin B expression in A375 cells (Figure 3g,h). These results suggest that ailanthone inhibits cell proliferation by arresting the cell cycle of the melanoma cells.

### 3.3. PI3K/Akt Signaling Is Involved in Ailanthone-Induced Cell Cycle Arrest in Melanoma B16 and A375 Cells

Considering that the PI3K/Akt signaling pathway plays an important role in cell cycle progression, the protein expression and phosphorylation levels of PI3K and Akt in melanoma cells were examined by Western blotting. We found that ailanthone remarkably reduced the expression levels of PI3K, p-PI3K, and p-Akt in B16 cells when compared to the control (Figure 4a,b). Ailanthone also significantly decreased the expression levels of PI3K, p-PI3K, and p-Akt in A375 cells relative to the control (Figure 4c,d).

### 3.4. Ailanthone Induces Cell Apoptosis in Melanoma B16 and A375 Cells

We also examined the morphologic changes in ailanthone-treated B16 and A375 cells using Hoechst 33258 staining. Compared to the control, distinct apoptotic characteristics such as nuclear condensation, irregular contraction of chromatin, and apoptotic bodies were observed in the ailanthone-treated B16 cells using a fluorescence microscope (Figure 5a). Flow cytometry analysis further showed that ailanthone significantly increased the apoptotic rate in a dose-dependent manner (Figure 5b,c). In addition, the above apoptotic characteristics were also detected in ailanthone-treated A375 cells using Hoechst 33258 staining (Figure 5d). Moreover, the apoptotic rates in ailanthone-treated A375 cells were significantly higher than those in the control (Figure 5e,f).

### 3.5. Ailanthone Induces Melanoma Cell Apoptosis Via A Caspase-Dependent Mechanism

As our results confirmed that ailanthone induced cell apoptosis in B16 and A375 cells, we next determined whether ailanthone regulated the expression levels of cell apoptosis-related proteins. Western blot analysis showed that the levels of caspase-9, cleaved caspase-9, and cleaved caspase-3 were upregulated, whereas caspase-3 was downregulated in ailanthone-treated B16 cells (Figure 6a,b). Ailanthone also upregulated caspase-9, cleaved caspase-9, and cleaved caspase-3 and downregulated caspase-3 in A375 cells compared to the control (Figure 6c,d).

### 3.6. Ailanthone Induces Melanoma Cell Apoptosis Via A Mitochondria-Mediated Signaling Pathway

Apoptosis is often accompanied by a decrease in mitochondrial membrane permeabilization [21]. A mitochondrial membrane potential measurement was conducted to confirm whether the mitochondria-mediated signaling pathway was involved in ailanthone-induced apoptosis. Mitochondrial membrane potential was measured with the membrane potential-sensitive dye JC-1 after ailanthone treatment. We observed a significant increase in the intensity of the green fluorescence in ailanthone-treated B16 cells, indicating that the mitochondrial membrane potential decreased after ailanthone treatment (Figure 7a). Western blot analysis showed that the level of cytoplasmic cytochrome c increased in the ailanthone-treated B16 cells (Figure 7b,c). Moreover, the levels of Apaf-1 and Bax significantly increased, whereas that of Bcl-2 significantly decreased in ailanthone-treated B16 cells relative to the control (Figure 7b,c). Similar results were observed in ailanthone-treated A375 cells. We detected a significant decrease in mitochondrial membrane permeabilization, a significant increase in the levels of cytoplasmic cytochrome c, Apaf-1, and Bax, and a significant decrease in the expression of Bcl-2 in the ailanthone-treated A375 cells relative to the control (Figure 7d,f). These results indicate that ailanthone induced cell apoptosis in melanoma B16 and A375 cells via the mitochondria-mediated apoptotic signaling pathway.

## 4. Discussion

The compound ailanthone isolated from the Chinese plant *A. altissima* has been shown to possess anti-tumor activity [11]. One ailanthone derivative SUN2071 with 15 beta-acyloxy side chain showed significant tumor growth inhibition against melanoma B16 cells [23]. However, the anti-tumor activity of ailanthone on melanoma and its mechanism of action have not been clarified. In this study, we found that ailanthone significantly suppressed cell viability and cell colony formation in B16 and A375 cells in a concentration-dependent manner.

Cancer is associated with uncontrolled cell proliferation, and the majority of drugs achieve antitumor effects by inhibiting uncontrolled cell proliferation by arresting the cell cycle of tumor cells [24]. There are four cell cycle regulatory points in the G1, S, G2, and M phases that can regulate cell cycle progression [25]. Ailanthone has been shown to exert anti-proliferative effects on Hun7 cells by blocking the cell cycle [15]. We further investigated whether ailanthone exerted anti-proliferative effects on B16 and A375 cells by triggering cell cycle arrest. In the present study, we found that the cell cycle progression of the B16 and A375 cells was blocked by ailanthone, and in turn, led to the inhibition of cell proliferation [26].

The p21 protein is a cyclin-dependent kinase inhibitor [27], and its downstream molecules cyclin E and cyclin B are involved in cell cycle progression at the G1/G2 phase [28]. Therefore, these proteins act as regulators of cell cycle progression [29]. In our study, we found that ailanthone upregulated p21 in both B16 and A375 cells and downregulated cyclin E in the B16 cells and cyclin B in the A375 cells. These findings indicate that ailanthone treatment induces cell cycle arrest in melanoma cells by regulating the expression of the cells’ cycle-related proteins. Ailanthone induced B16 cell cycle arrest at the G0/G1 phase and induced A375 cell cycle arrest at the G2/M phase. Further studies exploring the cell cycle distribution in ailanthone-treated B16 and A375 cells are warranted.

The PI3K/Akt signaling pathway has been associated with carcinogenesis [30]. Since the PI3K/Akt pathway, an important upstream factor of the DNA damage monitoring point [31], is a key regulator of cell survival and cell cycle in a variety of cancers [32], the activation of the PI3K/Akt pathway accelerates cell cycle progression [33]. Thus, to explore whether this signaling pathway is involved in the cell cycle arrest of ailanthone-treated B16 and A375 cells, we performed a series of Western blot assays. The results showed a decrease in the expression of PI3K and p-PI3K in the B16 and A375 cells after ailanthone treatment. Akt is one of the executors of PI3K that promotes cell growth [34]. Since the phosphorylation at Thr308 is necessary for the activation of Akt [35], the expression of p-Akt (Thr308) was also investigated. Ailanthone treatment resulted in a significant decrease in p-Akt expression, whereas no change in Akt expression was observed in both the B16 and A375 cells. Treatment of B16 and A375 cells with ailanthone resulted in a significant inhibition of the activation of the PI3K/Akt pathway, which in turn blocked mitotic onset [33]. These findings confirm that PI3K-Akt signaling is involved in ailanthone-induced B16 and A375 cell cycle arrest.

The occurrence of tumors is not only related to the uncontrolled proliferation of cells, but also to abnormalities of apoptosis [36]. Therefore, enhanced apoptosis is regarded as a potential method for cancer treatment. As ailanthone induces apoptosis in human NSCLC cells [14], we hypothesized that apoptosis also played a crucial role in ailanthone-treated B16 and A375 cells. The results of the Hoechst 33258 staining showed that ailanthone treatment of B16 and A375 cells induced nuclear condensation or granular fluorescence, which are typical features of apoptosis [16]. Meanwhile, the cell apoptosis rate of ailanthone-treated B16 cells measured by flow cytometry confirmed our previous results. The results of this study demonstrate that the anti-cancer effect of ailanthone on B16 and A375 cells is due in part to the induction of apoptosis.

Apoptotic cell death is dependent on members of the caspase family, which can cause a cascade that leads to cell death [37]. Caspases are central to the mechanism of apoptosis, which are both the initiators and executors of cell death [38]. Activation of caspase is considered as a typical marker of apoptosis [39]. We have found that ailanthone upregulates caspase-9 and cleaved caspase-9, which are primarily responsible for the initial steps of the apoptotic pathway [40] as well as the cleavage of cellular components [40]. Taken together, our results indicate that ailanthone induces apoptosis via a caspase-dependent mechanism.

Mitochondria play a central role in apoptotic cell death, which is mediated by outer membrane permeabilization in response to death triggers such as DNA damage and growth factor deprivation [41]. The decrease in mitochondrial membrane permeabilization is widely regarded as one of the earliest events of apoptosis [42]. In our study, we measured the changes in mitochondrial membrane potential using JC-1. Fluorescence microscopy showed that the proportion of green fluorescence in the B16 and A375 cells treated with ailanthone significantly increased, indicating that the mitochondrial membrane potential was significantly lower when compared to the control. The continuous reduction in the mitochondrial transmembrane potential will lead to the release of cytochrome c into the cytoplasm [43]. Cytochrome c that is released from the mitochondria then combines with Apaf-1 and caspase-9 to form a complex [44], Apaf-1 activates caspase-9 by interacting with CARD-CARD, and caspase-9 activates the downstream executor caspase-3 for the cleavage of cellular substrates, which in turn leads to apoptotic cell death [45]. In this study, we found that ailanthone induced an increase in the levels of cytoplasmic cytochrome c and Apaf-1 and subsequently activated caspase-9 and caspase-3, leading to mitochondria-mediated cell apoptosis.

Studies have shown that members of the Bcl-2 family of proteins play key roles in controlling the mitochondrial pathway [46,47], which has been shown to be one of the components of the mitochondrial permeability transition pore (mPTP) [48]. The effect of Bcl-2 depends on the ratio of its expression to Bax, which determines whether a cell undergoes apoptosis or survival upon stimulation with this signal. A reduction in the ratio of Bcl-2/Bax proteins indicates an alteration of the structure and permeability of the mitochondrial permeability transition pore, thereby causing mitochondrial-mediated death [49]. The protein expression levels of Bcl-2 and Bax were detected by Western blot analysis, which showed that the expression of Bax significantly increased and that of Bcl-2 significantly decreased after treatment with ailanthone. These findings indicate that ailanthone can reduce the permeability of the mitochondrial permeability transition pore (mPTP) by inhibiting the expression of Bcl-2 and increasing the expression of Bax [50], thereby promoting the formation of a complex of cytochrome c and Apaf-1 and activating caspase-9 and caspase-3, which is the cascade reaction that induces apoptosis. These findings clearly indicated that the mechanism of ailanthone-induced apoptosis in B16 and A375 cells involves the mitochondria-mediated apoptotic signaling pathway, which is regulated by the Bcl-2 family.

Bax and Bcl-2, which regulate apoptosis, are also important downstream factors of the PI3K/Akt pathway. The activation of Akt further triggers downstream factors such as the bcl-2 family [51]. The activation of PI3K-dependent Akt can depolymerize Bad and Bcl-2, and free Bcl-2 inhibits apoptosis [39]. Ailanthone treatment led to the downregulation of pro-apoptotic protein Bcl-2 and the upregulation of the anti-apoptotic protein Bax in B16 cells and A375 cells. These results indicate that the PI3K/Akt signaling pathway is also involved in mitochondria-mediated cell apoptosis in ailanthone-treated B16 and A375 cells.

However, the safety concerns of ailanthone should be noted. The anti-tumor effects of ailanthone were examined in melanoma A375 and B16 cells, but the cytotoxicity of ailanthone in normal cells, for example, human HaCaT keratinocytes or mouse L929 fibroblasts were not determined. A recent study demonstrated that ailanthone significantly blocks tumor growth and metastasis, and does not exert obvious hepatotoxicity in prostate cancer 22RV1 tumor-bearing mice [52], implying that ailanthone could be a potential candidate for cancer treatment.

## 5. Conclusions

The present study has shown that ailanthone inhibits cell proliferation in B16 and A375 cells via the PI3K-Akt signaling pathway and induces cell apoptosis via the mitochondria-mediated signaling pathway. This study reveals that ailanthone may be potentially utilized as an anti-tumor agent in the management of malignant melanoma.

## Figures and Tables

**Figure 1:** The structure of ailanthone.

**Figure 2:** Ailanthone inhibits cell proliferation and cell colony formation in melanoma B16 and A375 cells. (**a**) After treatment with different concentrations of ailanthone (0.25, 0.5, 1, 2, 4, 8, and 16 μM) for 24 h, the cell viabilities of B16 and A375 cells were determined using the cell counting kit-8 assay. (**b**) Statistical analysis of the number of cell colonies in ailanthone-treated B16 and A375 cells. (**c**) The cell colonies were stained with crystal violet and observed under an inverted microscope. The data are presented as the mean ± SD (*n* = 3). * *p* < 0.05, ** *p* < 0.01 compared with the control B16 cells. ^#^ *p* < 0.05, ^##^ *p* < 0.01 compared with the control A375 cells.

**Figure 3:** Ailanthone induces cells cycle arrest and regulates cell cycle-related proteins in melanoma B16 and A375 cells. (**a**) Cell cycle distributions of the B16 cells were measured by flow cytometry after treatment with various concentrations of ailanthone for 24 h. (**b**) Statistical analysis of the cell cycle distribution of ailanthone-treated B16 cells. * *p* < 0.05, ** *p* < 0.01 compared with the control B16 cells. (**c**) The levels of p21 and cyclin E in ailanthone-treated B16 cells were examined by Western blotting. (**d**) Quantitative analysis of the levels of p21 and cyclin E in ailanthone-treated B16 cells. * *p* < 0.05, ** *p* < 0.01 compared with the control B16 cells. (**e**) Cell cycle distribution of the A375 cells was measured by flow cytometry after treatment with various concentrations of ailanthone for 24 h. (**f**) Statistical analysis of cell cycle distributions of the ailanthone-treated A375 cells. ^#^ *p* < 0.05, ^##^ *p* < 0.01 compared with the control A375 cells. (**g**) The levels of p21 and cyclin B in ailanthone-treated A375 cells were examined by Western blotting. (**h**) Quantitative analysis of the levels of p21 and cyclin B in ailanthone-treated B16 cells. ^#^ *p* < 0.05, ^##^ *p* < 0.01 compared with the control A375 cells. The data are presented as the mean ± SD (*n* = 3).

**Figure 4:** PI3K-Akt signaling is involved in the cell cycle arrest of ailanthone-treated melanoma B16 and A375 cells. (**a**) The levels of p-PI3K, PI3K, p-Akt, and Akt in ailanthone-treated B16 cells were examined by Western blotting. (**b**) Quantitative analysis of the levels of p-PI3K, PI3K, p-Akt, and Akt in ailanthone-treated B16 cells. * *p* < 0.05 compared with the control B16 cells. (**c**) The levels of p-PI3K, PI3K, p-Akt, and Akt in ailanthone-treated A375 cells were examined by Western blotting. (**d**) Quantitative analysis of the levels of p-PI3K, PI3K, p-Akt, and Akt in ailanthone-treated A375 cells. ^#^ *p* < 0.05, ^##^ *p* < 0.01 compared with the control A375 cells. The data are presented as the mean ± SD (*n* = 3).

**Figure 5:** Ailanthone induces cell apoptosis in melanoma B16 and A375 cells. (**a**) Representative morphological images of ailanthone-treated B16 cells after Hoechst 33258 staining. (**b**) The apoptotic rates of ailanthone-treated B16 cells were measured by flow cytometry. (**c**) Quantitative analysis of the apoptotic rates of ailanthone-treated B16 cells. **p < 0.01 compared with the control B16 cells. (**d**) The representative morphological images of ailanthone-treated A375 cells after Hoechst 33258 staining. (**e**) The apoptotic rates of ailanthone-treated A375 cells were measured by flow cytometry. (**f**) Quantitative analysis of the apoptotic rates of ailanthone-treated A375 cells. ^##^ *p* < 0.01 compared with the control A375 cells. The data are presented as the mean ± SD (*n* = 3).

**Figure 6:** Ailanthone induces melanoma cell apoptosis in a caspase-dependent mechanism. (**a**) The expression levels of caspase-9, cleaved caspase-9, caspase-3, and cleaved caspase-3 in ailanthone-treated B16 cells were examined by Western blotting. (**b**) Quantitative analysis of the expression levels of caspase-9, cleaved caspase-9, caspase-3, and cleaved caspase-3 in ailanthone-treated B16 cells. * *p* < 0.05, ** *p* < 0.01 compared with the control B16 cells. (**c**) The expression levels of caspase-9, cleaved caspase-9, caspase-3, and cleaved caspase-3 in ailanthone-treated A375 cells were examined by Western blotting. (**d**) Quantitative analysis of the expression levels of caspase-9, cleaved caspase-9, caspase-3, and cleaved caspase-3 in ailanthone-treated A375 cells. ^#^ *p* < 0.05 compared with the control A375 cells. The data are presented as the mean ± SD (*n* = 3).

**Figure 7:** Ailanthone induces cell apoptosis in melanoma cells via the mitochondria-mediated apoptotic signaling pathway. (**a**) Changes in mitochondrial membrane permeabilization in ailanthone-treated B16 cells was observed by fluorescence microscopy. (**b**) The expression levels of cytoplasmic cytochrome C, Apaf-1, Bcl-2, and Bax in ailanthone-treated B16 cells were examined by Western blotting. (**c**) Quantitative analysis of the levels of cytoplasmic cytochrome C, Apaf-1, Bcl-2, and Bax in ailanthone-treated B16 cells. * *p* < 0.05 compared with the control B16 cells group. (**d**) Changes in mitochondrial membrane permeabilization in ailanthone-treated A375 cells were assessed by fluorescence microscopy. (**e**) The expression levels of cytoplasmic cytochrome C, Apaf-1, Bcl-2, and Bax in ailanthone-treated A375 cells were examined by Western blotting. (**f**) Quantitative analysis of the levels of cytoplasmic cytochrome C, Apaf-1, Bcl-2, and Bax in ailanthone-treated A375 cells. ^#^ *p* < 0.05, ^##^ *p* < 0.01 compared with the control A375 cells. The data are presented as the mean ± SD (*n* = 3).
